# Review on Comfort Nursing Interventions for Patients Undergoing Neurosurgery and General Surgery

This article has been retracted.

**DOI:** 10.1155/2022/6735054

**Published:** 2022-08-10

**Authors:** Limin Wu, Yingfa Chen, Jin Zhang, Honglan Yu

**Affiliations:** ^1^Department of General Surgery, No. 1128, Dacheng, Anzhen, Xishan, Wuxi, Jiangsu, China; ^2^Department of Neurology, Wuxi Xishan People's Hospital, No. 1128, Dacheng, Anzhen, Xishan, Wuxi, Jiangsu, China

## Abstract

**Objective:**

To summarize the commonalities and particularities of comfort care interventions for neurology and general surgery patients.

**Methods:**

The development of comfort care and its practical application in neurology and general surgery were discussed and summarized by searching the current literature on comfort care interventions for neurology and general surgery patients, including case reports, clinical studies, and systematic reviews.

**Results:**

Comfort nursing intervention is a kind of nursing intervention with integrity and creativity. In addition to its uniqueness, the comfort nursing model also has strong effectiveness. Clinical holistic nursing has been significantly improved through the application of comfort nursing intervention theory, and its nursing mode has enhanced the connotation of clinical nursing.

**Conclusion:**

Comfort nursing intervention for neurology and general surgery patients can help patients recover and deserves further promotion.

## 1. Introduction

Neurology is a secondary discipline within clinical neurology. There are many diseases that are treated in its department, and the majority of patients are elderly [1]. It is common that elderly patients in neurology, due to the influence of illness or age, will suffer from different degrees of hemiplegia, aphasia, confusion, etc. It is clinically necessary to develop neurological care in a precise and comfortable manner to help patients recover and improve their quality of life [2]. General surgery is the largest specialty within the surgical system, and it is a clinical discipline with surgery as its primary modality of treatment. As surgical patients are usually in critical condition, and patients in their departments present a variety of nursing risks, it is difficult to provide nursing care. The continuous improvement in people's income and clinical medical level in China has led to an increase in the demand for clinical care. The comfort nursing intervention is an exceptional, creative, and holistic nursing approach, and the effectiveness of its nursing model has been recognized by a number of departments. Almost all patients may create a pleasant condition with this mode, and its application can successfully lessen or alleviate the discomfort of patients during treatment [3].

To date, the concept of patient-centered holistic nursing has gradually become a consensus in the industry, and the proposal and application of comfort nursing intervention theory has enriched the meaning of clinical nursing. In addition, with the development of modern medical model, the theoretical system of modern nursing has deepened the connotation of nursing service and expanded the scope of nursing service. Under the new historical conditions, traditional Chinese medicine (TCM) nursing has exhibited a certain advantage; people have a new understanding of TCM nursing technology and rationally apply it to the condition observation, emergency treatment, and psychological care of emergency patients. Therefore, TCM nursing is also helpful for the recovery of patients after neurology and general surgery [4]. The purpose of this review was to analyze, synthesize, and explore the commonalities and specificities of comfort care interventions applied to neurology and general surgery patients.

## 2. Progress of Comfort Nursing

### 2.1. Comfort Nursing Theory: Its Emergence and Improvement

According to Miss Nightingale, the founder of nursing education, the patient's ward should have several aspects such as cleanliness, comfort, quietness, and a pleasant fragrance, which is the foundation of comfort nursing theory. According to Kolcaba [5], the theoretical framework for comfort nursing was formally formulated in 1995. Kolcaba believed that comfort nursing is the inevitable outcome of the entire nursing process. The double-C nursing model was also proposed by Hiao Fufeng from Taiwan in 1998, who believes that nursing research and practice should be focused on the comfort of patients. According to Hiao's double-C nursing model, “double-C” refers to “nursing activities + comfort activities.” Nursing activities refer to taking care of patients, including providing simple comfort care; comfort activities pertain to enabling patients to achieve physiological, psychological, and spiritual comfort.

### 2.2. Connotation Policy for Comfort Nursing Services

The connotation of comfort nursing is to enable the patient to obtain a pleasant state in terms of psychology, physiology as well as soul. This will include

#### 2.2.1. Psychological Care

In the event of a disease, the patient will learn from a familiar situation when they are afflicted. However, the environment changes into an unfamiliar one. As a result of the unfamiliar environment, the psychological state of the patient will cause a certain amount of anxiety, and the comfort nurse shall present a dignified appearance and decent language in order to ease the patient's fears. Comfort enables the patient to form a bond of trust with the nursing staff in a short period of time, which helps to make the patient's mind and body happy, which helps to make the patient's mind comfortable as well. It is the comfort nurses' responsibility to welcome patients and introduce them patiently to the competent doctors, nurses, ward environment, rules, and regulations, as well as work procedures related to their diseases, in order to help the patients adapt to the hospital environment. According to Li Song and others, a cup of hot water, a greeting, a smile, etc., can greatly relieve the tension of patients and reduce the distance between nurses and patients. In the course of the nursing process, nurses should listen more and respect the opinions and suggestions of patients [6].

#### 2.2.2. Physical Comfort Nursing

The purpose of comfort nursing is to provide a clean, comfortable, quiet, and clutter-free medical environment for the patient and to adjust the lighting, temperature, and humidity in the patient's room to a comfortable and appropriate level. The staff may also provide humorous books, healthy and nutritious recipes, and fashion magazines for the patients or play some relaxing music for them, all of which can help the patients distract themselves from their discomfort. A stable mood is conducive to the health of the patient's body and mind. Additionally, nurses will provide patients with information regarding complications and skin-related comfort measures. Nurses should pay close attention to the essentials of fast, stable, and accurate care when implementing nursing procedures, grasp the appropriate nursing intensity, and strive to minimize patient discomfort.

#### 2.2.3. Mental Comfort Nursing

The comfort nursing staff will be aware of the patient's beliefs and will respect and support those beliefs. It is the responsibility of nursing staff to take the initiative to understand some of the patient's preferences and to aid the patient's preferences, entertainment, and learning, assisting patients as they explore the meaning of life. As well as encouraging good relationships between patients and other patients, nursing staff will also ask family members to encourage and support patients. It is necessary to make patients feel wanted and needed in order to reduce their loneliness, to make them appreciate life [7].

### 2.3. Different Types of Comfort Care

Comfort care can be divided into two types: basic comfort care and advanced comfort care.

1. The basic comfort care guidelines are primarily based on common sense, such as avoiding noise after the patient has fallen asleep and paying attention to the warm environment when checking the patient's physical condition. It is not typically necessary to perform detailed demonstrations and research in order to provide comfort care.
2. Advanced comfort care is usually above common sense in everyday living, and it is typically divided into two categories: invasive and noninvasive. Invasive care includes methods for administering anesthesia, taking blood, and administering medications in a comfortable manner [8]. On the other hand, noninvasive care involves psychological, physical, social, and spiritual comfort. Nursing students are required not only to acquire basic medical knowledge and nursing professional knowledge but also to actively get involved in related fields such as psychology, pharmacology, and traditional Chinese medicine so that they can provide better comfort care to patients.

### 2.4. Advances in Clinical Practice and Application of Comfort Nursing

1. A comfort nurse's primary responsibility is to provide a quiet, clean, and comfortable environment for patients. It was pointed out by the scholar Li Ming and others that comfortable temperature, humidity, smell, etc., can play a significant role in patients' physical and mental well-being and their ability to recover. Comfort nursing can make the patient's body and mind achieve the best state, which has a very important impact on the patient's follow-up treatment effect [9].
2. The diagnosis and treatment technology of comfort nursing will run throughout the daily life of the patient, as well as into the details of the patient's daily care. When it comes to clinical nursing behaviors, skilled operations, sufficient knowledge, and warm service are the most important guarantees for a comfortable nursing experience. Currently, the clinical needs for nursing and the research on nursing innovation give more consideration to the comfort effect. The purpose of comfort nursing is to minimize the patient's pain, anxiety, and other physical and psychological discomfort, regardless of the prognosis of the patient's disease [10].
3. To date, the theory of comfort nursing has been constantly revised and improved, but its enthusiasm and sustainable development have not been replicated. As a patient-centered, patient-oriented, selective nursing method, comfort nursing has long valued the comfort effect felt by the patient as its primary goal, which allows its various aspects to work together harmoniously. Despite its simplicity and operability, comfort nursing has strong connection between clinical nursing practice and nursing research, and it has been shown to significantly improve the quality of clinical nursing. The reason is that its theory is in accordance with holistic nursing and evidence-based nursing. Since comfort nursing has rich connotations, it requires nursing staff to broaden their knowledge. This encourages clinical nursing staff to learn relevant knowledge, in order to be able to meet the increasing comfort needs of patients in the future. Several nursing experts with their own strengths have laid the foundation for improving the status of clinical nursing [11].
4. Comfort nursing understands that even if a patient's body is afflicted with disease, he or she remains a social being with his or her own personality, so his or her dignity cannot be dismissed. The nursing staff should treat the patient with the utmost respect, which is reflected in the quality of the patient's life. Clinical treatment and nursing are intended not only to treat the patient's physical illness but also to prevent the disease process, prolong the patient's life, and at the same time respect the patient's wishes. In addition to encouraging patients to fulfill their own wishes, the nursing staff should consider using life support technology when necessary to make up for the deficiencies of traditional concepts.

### 2.5. Chinese Medicine Nursing

1. Observing the condition: The human body is an organic whole, and local lesions can affect the whole body; internal organs lesions can be reflected from various aspects such as the head, face, facial features, and four limbs. And the four diagnostic methods of TCM: Wang (seeing), Wen (listening and smelling), Wen (questioning), and Qie (touching pulses) advocated by Chinese medicine are favorably in tune with this [12]. In emergency care, rhubarb can be used as a catharsis for the care of patients with acute poisoning to help the patient to eliminate the poison; for some common multiple diseases, bupleurum injection and scraping can be used for routine care; in addition, during first aid, the corresponding acupoints can be stimulated for adjuvant therapy [13].
2. First aid: TCM nursing techniques are relatively simple and easy to master and can effectively deal with patients' emergencies in the process of practical operation. In addition, using the knowledge of TCM to observe the changes of the patient's complexion and tongue coating can help to indicate the patient's condition changes. If the patient's tongue and pulse change significantly, such as the red tongue turning into a red-purple tongue, it represents that the evil has entered the blood, indicating a critical condition [14, 15].
3. Emotional care: Clinical practice shows that the more serious the patient is, the more emotional the patient is, and the high-risk disease brings huge psychological pressure to the patient [16]. Emotional nursing occupies an important position in TCM nursing. If the emotions are too stimulated, the internal organs will be affected. In the case of imbalance of yin and yang, the dysfunctions of the internal organs are caused. TCM nursing focuses on the methods of enlightenment, diversion, and suggestion to smoothen the qi of patients [17].
4. Dietary care: TCM should not use all drugs in the nursing process because drugs often damage the vitality of the human body after reaching a certain amount [18]. TCM believes that food and medicine should be combined. Nursing staff can give corresponding dietary guidance based on the principles of TCM such as “Yang should be cultivated in spring and summer, and Yin in autumn and winter” and the patient's condition. Scientific and reasonable collocations need to be carried out according to the climate, the patient's condition, and the nature of the food, so as to reduce the stimulation of the diet to the patient [19, 20].

## 3. Application and Specific Measures of Comfort Nursing in Neurology and General Surgery Departments

### 3.1. The Application and Specific Measures of Comfort Nursing in the Neurology Department

The application of comfort nursing in the neurology department should reflect its “people-oriented” philosophy and should adhere to all patient-centered nursing concepts in order to implement effective and humanized nursing measures that can provide neurological benefits for patients. It should establish a solid foundation for the treatment and rehabilitation of medical patients. Patients in the neurology department are prone to tension, irritability, low self-esteem, fear of dragging family members, and other emotions as a result of their paralysis and the loss of their self-care abilities and language abilities [21], which makes them susceptible to anxiety, tension, and irritability [22]. These negative emotions will often lead patients to give up their treatment.

Comfort nurses who work in the neurology department communicate well with patients and provide them with appropriate psychological counseling and psychological counseling in a timely manner. A comfortable nurse will look at the issue from the point of view of the patient, will understand the patient's pain, and will provide comfort and encouragement to the patient in time, which will enable the patient's underlying negative emotions to vent and be relieved, and in turn, will improve their psychological state. Having a comfortable environment allows patients to remain in a positive frame of mind during future treatment [23]. Patients with neurology problems often require prolonged bed rest and suffer from urinary incontinence, causing psychological and physiological distress to the patient. Thus, the nursing staff will regularly assist the patient in changing their bed position, thereby reducing the risk of the patient's failure. Furthermore, the comfort caregiver provides skin comfort care, which contributes to maintaining the integrity of a patient's skin. Comfort nurses are responsible for aiding patients with breathing, digestion, excretion, sleep, rest, and disinfecting and isolating patients to prevent cross-infections [24].

### 3.2. The Practical Application and Specific Measures of Comfort Nursing in General Surgery

Comfort nursing formulates different nursing measures based upon the surgical procedure and the part of the patient that requires care. Comprehensive overall comfort nursing, including different comfort nursing measures before, during, and after the operation are the main measures.

1. The purpose of preoperative comfort nursing is to help patients relax, adjust their diet, assist them in preparing for surgery, and provide information related to health care before and after surgery [25].
2. The nursing care in the intraoperative period includes pacification of patients, reducing anxiety, and increasing patients' confidence in the treatment; adjusting the temperature and humidity in the operating room; and aiding the patient to situate themselves in a comfortable and stable position during surgery to reduce the physiological discomfort caused by the operation. The nursing staff should be steady, accurate, and light when performing various procedures. An efficient nursing staff should be technically skilled and standardized and strive to prevent the adverse stimulation and unnecessary pain caused by careless or repeated operation. During the operation, the nursing staff should check closely for abnormalities in the patient's vital signs and puncture site [26].
3. Preoperative comfort nursing interventions are designed to reduce the pain and stress response of the patient and to prevent sharp fluctuations in their vital signs.

The nursing staff must closely observe the postoperative complications of the patients, report any problems in a timely manner, and cooperate with the doctors in the treatment of the patients.

Nurses should recognize the psychological needs of patients after surgery and provide targeted psychological counseling to assist in the early recovery of patients [27].

## 4. Common Characteristics of Comfort Nursing for Neurology and General Surgery Patients and Particular Characteristics of Comfort Nursing for Neurology and General Surgery Patients

### 4.1. The Commonness of Comfort Nursing for Patients in Neurology and General Surgery

Currently, clinical nursing work focuses primarily on neurology and general surgery. The comfort nursing approach is commonly used within these departments [28]. In general, neurology patients have varying degrees of paralysis, aphasia, and self-care ability. There is a low level of emotional maturity, etc., which can lead to irritability, low self-esteem, fear, depression, self-defeating behavior, and other adverse effects. General surgery patients usually undergo surgical treatment. As an invasive procedure, surgical treatment will also have adverse effects on the patient's heart, as well as possible complications after surgery. This condition is accompanied by severe pain, which further affects the patient's mood [29].

Accordingly, this study concludes that the commonality in patient care between neurology and general surgery lies in the psychological component of comfort care. Despite the fact that patients in the two departments have experienced different adverse emotions, both departments require comfort care; this includes psychological support. A comfortable psychological nursing approach refers to a series of nursing interventions, such as voice communication and behavioral guidance, that are intended to alleviate patients' negative emotions. Studies by scholars such as Ma Wenli have indicated that comfort nursing interventions can contribute to a more comfortable psychological state for the patient. It has been shown that a comfortable psychological state can significantly improve both patient enthusiasm for treatment and its effectiveness [30].

### 4.2. The Particularities of Comfort Nursing for Patients in Neurology and General Surgery

There are some particulars concerning the nursing care provided to patients in the Department of Neurology and General Surgery. Nursing in the Department of Neurology is unique in the sense that patients in the Department of Neurology undergo a long-term treatment and rehabilitation process. These patients require long-term hospitalization. It is common for patients in the Department of Neurology to have strong feelings and thoughts, such as loneliness and helplessness, during the course of their treatment. The subjective emotional aspects of these patients will significantly affect their follow-up treatment and recovery, so comfort nursing for neurology patients is primarily based on companionship, care, and careful attention.

Nursing care for general surgery patients is distinguished by the fact that they do not need long periods of rehabilitation treatment. The discomfort they experience in their bodies is caused by the invasive nature of the surgical procedure and its potential complications. For general surgery patients, the focus of comfort nursing care will be on timely postoperative analgesia, strengthening the patient's nutrition intake, and assisting the patient in accelerating their body's recuperation process [31].

However, we only included the application in neurology and general surgery in this study. In the future, we would include more departments to enrich its value; second, we only qualitatively described and reviewed the previous studies. Future studies using a quantitative method are warranted to more accurately assess its value.

## 5. Conclusion

In conclusion, when comfort nursing intervention is used in patients with neurology and general surgery, it fully embodies the comprehensive nursing concept of individual care, disease care, and need care. As a result, comfort nurses must continually develop their cultural literacy and their ability to communicate, observe, analyze, and solve problems along with establishing good patient relationships; only in this manner can they provide patients with a more comfortable experience. Despite the fact that the comfort nursing model still has certain shortcomings and imperfections, a healthy development of its nursing model will have a significant impact on the field of clinical nursing and in-depth nursing research; the positive impact will be immeasurable.

## Data Availability

No data were used to support this study.
